# Amelioration of Auditory Response by DA9801 in Diabetic Mouse

**DOI:** 10.1155/2015/230747

**Published:** 2015-03-24

**Authors:** Yeong Ro Lee, Bin Na Hong, You Ri Her, Rodrigo Castañeda, Hyo Won Moon, Tong Ho Kang

**Affiliations:** ^1^Graduate School of Biotechnology, Kyung Hee University, Global Campus, Gyeonggi 446-701, Republic of Korea; ^2^Department of Oriental Medicinal Materials & Processing, College of Life Sciences, Kyung Hee University, Global Campus, Gyeonggi 446-701, Republic of Korea; ^3^Department of Audiology, Nambu University, Gwangju 506-824, Republic of Korea

## Abstract

Diabetes mellitus (DM) is a metabolic disease that involves disorders such as diabetic retinopathy, diabetic neuropathy, and diabetic hearing loss. Recently, neurotrophin has become a treatment target that has shown to be an attractive alternative in recovering auditory function altered by DM. The aim of this study was to evaluate the effect of DA9801, a mixture of *Dioscorea nipponica* and *Dioscorea japonica* extracts, in the auditory function damage produced in a STZ-induced diabetic model and to provide evidence of the mechanisms involved in enhancing these protective effects. We found a potential application of DA9801 on hearing impairment in the STZ-induced diabetic model, demonstrated by reducing the deterioration produced by DM in ABR threshold in response to clicks and normalizing wave I–IV latencies and Pa latencies in AMLR. We also show evidence that these effects might be elicited by inducing NGF related through Nr3c1 and Akt. Therefore, this result suggests that the neuroprotective effects of DA9801 on the auditory damage produced by DM may be affected by NGF increase resulting from Nr3c1 via Akt transformation.

## 1. Introduction

Diabetes mellitus (DM) is one of the most common metabolic diseases and is divided according to the mechanism in which the hyperglycemia is generated into two types, dysfunction in insulin secretion and resistance to its activity. This disruption in metabolism involves the development of many disorders in the entire organism, such as retinopathy, neuropathy, and nephropathy. Recently, evidence studies reported that hearing impairment could be caused by DM [1]. DM induces cochlear dysfunction by loss of outer hair cells (OHCs) and spiral ganglion neuron atrophy, degeneration of the cochlear lateral walls in the inner ear [2–7], because high glucose level may alter inner ear function by affecting the inner ear damage through sorbitol pathway involvement and accumulation of advanced glycation end products. Furthermore, the hyperglycemic state produced in DM has been related to hearing impairment in a short period disruption in auditory storage and slow speed of auditory information processing [8–10]. These failures are accompanied by an enhanced rate of programmed cell death, or apoptosis in the auditory system. In addition, our previous study concluded that hearing impairment was found in the streptozotocin- (STZ-) induced diabetic mouse model, developing an impairment in the auditory pathway from the auditory nerve to the midbrain [11].

NGF is essential for viability, differentiation, and maintenance of nerve cells [12, 13]. Also, it contributes to repair the nervous system [14, 15]. NGF binds with two classes of receptors, a tyrosine kinase receptor (TrkA, TrkB, and TrkC) and a low-affinity receptor called p75^NTR^ [16–19]. It has been proposed that when NGF binds with Trk, it became phosphorylated itself, serving as a binding site for specific signaling protein such as Akt through PI3 kinase [20–24], which binds and phosphorylates Bad, a member of the Bcl-2 family [25–27], blocking the apoptosis pathway, resulting in increased cell viability. NGF has shown to be induced by glucocorticoid* in vivo* [28, 29]. In addition, Nr3c1 is glucocorticoid receptor which controls transcription of target genes, and expression was found in PC12 cell, mouse, rat, and human auditory system, and previous study reported that glucocorticoid sensitivity might be dependent on expression level of Nr3c1 [30–35].

Recently, pathogenetic control of diabetic neuropathy has been improved after neurotrophic therapy, such as NGF treatment, and by targeting pathological factors, in both STZ-induced DM animal models and in the human condition [36, 37], which could be relevant to diabetic hearing impairment. In diabetic neuropathy, NGF levels are decreased in peripheral nerve such as superior cervical ganglion and sciatic nerve in STZ-induced rats [38, 39]. It also may be involved in differentiation of acoustic ganglion cells and hair cells [40]. DA9801 has shown to induce endogenous NGF expression, supported by a recovery effect on the peripheral nerve* in vitro* and* in vivo* [41–44]. In our previous study of DA9801, a mixture of* Dioscorea japonica* and* Dioscorea nipponica* extracts showed a peripheral nerve protection effect in rats with STZ-induced diabetes through induction of endogenous NGF. In addition, other studies have confirmed the ameliorative effect of DA9801 on DPN in diabetic rats and even in a phase II clinical study, improving nerve conduction velocity and promoting recovery from neuronal degeneration [41–44]. The aim of the study was to evaluate the ameliorative effects produced by DA9801 on the auditory dysfunction produced in a STZ-induced diabetic model and to provide evidence of the possible mechanism of action in the auditory neural protection and survival related to induce endogenous NGF through Nr3c1.

## 2. Materials & Methods

### 2.1. Animal

All of the experimental procedures were performed in accordance with the Principles of Laboratory Animal Care (NIH publication, #80-23, revised 1996) and the Animal Care and Use Guidelines of Nambu University, Korea. Seven-week-old adult male ICR mice were obtained from Samtako Co. (Osan, Korea) with an average weight between 30 and 33 g. The mice were maintained in a standard laboratory animal facility at 12 h light/12 h dark cycles with food and water* ad libitum*.

### 2.2. Diabetes Mellitus Induction

DM was induced by a single 120 mg/kg I.P. injection of STZ dissolved in 0.01 M sodium citrate buffer (pH 4.5). One week later, blood glucose measurements from nonfasting mice were taken from mouse tail pricks with strip-operated blood glucose sensors (ONETOUCH Ultra, Inverness Medical Ltd., UK). Diabetic mice with blood glucose levels ≥300 mg/dL were used in experiments.

### 2.3. Plant Material and Extract Preparation

Dried rhizomes of* D. japonica* and* D. nipponica* were mixed in a specific ratio (3.5 : 1) and extracted with 50% ethanol three times at room temperature for 48 h. After filtration, the aqueous ethanol extract was evaporated under reduced pressure rotary vacuum evaporator with vacuum MZ 2C NT + AK + EK (Vacuubrand, Korea). The extract was then lyophilized for a complete removal of the residual solvent to yield a brown powder. The contents of two marker components, dioscin (1.37%) and allantoin (3.29%), in DA9801 were evaluated by HPLC.

### 2.4. DA9801 Administration

Animals assigned to the evaluation of the auditory function and NGF levels were divided into 3 groups (*n* = 10/group). Nondiabetic ICR mice (normal group) and nontreated STZ-induced diabetic mice (DM group) were treated orally once daily with 0.5 mL of distilled water, and treated STZ-induced diabetic mice (DM-DA) were treated orally with DA9801 100 mg/kg once daily for 8 weeks.

Animals assigned to the evaluation of the mechanisms related to NGF were divided into 3 groups (*n* = 5/group). Normal group mice were treated with 0.5 mL of distilled water and DA100 group and DA300 group mice were treated orally with 100 mg/kg and 300 mg/kg doses of DA9801.

### 2.5. Auditory Function Tests

To investigate the DA9801 effect on auditory impairment, hearing thresholds and latencies were measured in normal, DM, and DM-DA groups using auditory brainstem response (ABR) and auditory mid-latency response (AMLR). The auditory function tests were performed with the mice under anesthesia after an I.M. administration of xylazine (0.43 mg/kg) and ketamine (4.57 mg/kg). The rectal temperature was maintained at 37°C ± 0.5°C using a heating lamp at the time of testing.

For the auditory electrophysiological tests, two-channel recordings (GSI Audera, Viasys Healthcare Inc., USA) were obtained through needle electrodes inserted subcutaneously at the vertex. Reference electrodes were placed below the pinna of the left and right ears, and a ground electrode was inserted into the shoulder. Electrode impedances were in the range of 2 kΩ to less than 5 kΩ for the electrode pairs.

For the ABR recordings, alternating clicks (0.1 ms duration) were delivered through earphones (Etymotic ER-3A) at a rate of 20.1 stimuli/s. Physiological filters were set to pass electrical activity between 100 and 3000 Hz. Monaural responses were recorded for each mouse and averaged in a 10.24 ms time window. One thousand sweeps were collected. To determine the thresholds of ABR recordings, the clicks were reduced in 10 dB steps. When no response was detected, the level increased in 5 dB steps until a response was determined. ABR parameters were evaluated based on the hearing thresholds and interpeak latencies of waves I–IV at a peak sound pressure level (pSPL) of 90 dB.

For the AMLR measurements, rarefaction clicks (0.1 ms duration) were delivered through earphones at a rate of 9.1 stimuli/s. Filters were set to pass activity between 10 and 250 Hz. An average of 250 sweeps was determined in a 70 ms time window. The parameters of AMLR were evaluated with absolute latencies of wave Pa at a pSPL of 90 dB.

### 2.6. NGF Assays

In order to evaluate NGF level in peripheral nerve, after the final auditory function tests were taken 8 weeks after treatment, serum and sciatic nerves were collected for NGF evaluation. Tissue samples were homogenized in NGF lysis buffer (Tris–HCl 100 mM, bovine serum albumin (BSA) 2%, NaCl 1 M, EDTA–4Na 4 mM, Triton X-100 2%, sodium azide 0.1%, pH 7.0, and phenylmethylsulfonyl fluoride 17 *μ*g/mL) and centrifuged at 4°C and 14,000 rpm during 20 min. The supernatant was subjected to ELISA in 96-well plates as described elsewhere, following the manufacturer's instructions.

### 2.7. Total RNA Preparations

The nondiabetic ICR mice (normal) were treated once orally with 0.5 mL of distilled water with DA9801 at 100 and 300 mg/kg (DA100 and DA300). Liver tissues were collected after 2 hours of treatment. Total RNA was isolated from the liver using Trizol Reagent (Life science), following the manufacturer's instructions. 500 *μ*L of the Trizol reagent was added to tissue sample and was homogenized. In addition, 100 *μ*L of chloroform (Sigma) was added, and a vortex was used for 10–15 sec and then centrifuged at 14,000 rpm for 15 min at 4°C. After taking the supernatant, the same amount of isopropanol (JUNSEI) was added. Total RNA was transferred into a pellet and washed with 75% EtOH in DEPC treated water (Sigma). The amount of RNA was measured by NanoDrop 2000 (Thermo scientific).

### 2.8. Quantitative Real-Time PCR

In order to evaluate Nr3c1 and TrkA mRNA expression level the following was done First, DNase I (Promega) was used in order to digest genomic DNA. cDNA was synthesized from 4 mg of total RNA using the RevertAid First Strand cDNA Synthesis Kit (Thermo Scientific) and OligoDT primer, following the manufacturer's instructions. Each real-time PCR was carried out in triplicate in a total of 20 *μ*L reaction mixture in Rotor gene Q (Qiagen) using specific primer (Table 1). The housekeeping gene *β*-actin was concurrently amplified in each sample as a control and was used for normalization. The Ct (threshold cycle) values of target genes obtained from the liver samples from the DM and DA100 groups complemented line were normalized to the endogenous reference gene actin (ΔCt = Ct_target_ − Ct_reference_) and compared with those values obtained from the calibrator normal group (ΔΔCt = ΔCt_sample_ − ΔCt_calibrator_) [45].

### 2.9. Protein Extraction

Frozen liver tissue extraction samples were prepared by homogenization in 500 *μ*L of iced extraction buffer (HEPES 20 mM, KCl 100 mM, glycerol 5%, EDTA 5 mM, MgCl_2_ 1 mM, DTT 1 mM, and Triton X-100 0.1%) with protease inhibitors (Roche) and then centrifuged at 14,000 rpm at 4°C for 15 min, and the supernatant was collected in a new tube. The amount of protein was measured by NanoDrop 2000 (Thermo scientific). Then the same amount of 2X SDS-PAGE sample buffer (1 M Tris (pH 6.8), 0.5 M EDTA, 10% SDS, 2-mercaptoethanol, 50% glycerol, and bromophenol blue) was added to the extract of protein. The mixture was boiled at 95°C for 5 min and then kept at −20°C.

### 2.10. Western Blotting

The 40 *μ*g of total protein was loaded to the SDS-PAGE and subsequently transferred to nitrocellulose membrane. The membrane was blocked by 5% skim milk (Bio Basic Canada Inc.) or 5% BSA (Roche) with TBS-T. After blocking, the membrane was probed with dilution of the anti-Nr3c1 (Bethyl), anti-p-Akt (Cell Signaling), and anti-*β*-actin (Santa Cruz) primary antibody, followed by the addition of horseradish peroxidase- (HRP-) conjugated secondary antibody. Immunoreactive proteins were visualized using a WEST-One (iNtRON). Band intensities were determined using the ImageQuant LAS 4000 (GE Healthcare) and Quantity One software (Bio-Rad). *β*-actin was used as constitutive control for normalization.

### 2.11. Statistical Analysis

Data were analyzed using the Prism 5 Statistical Software package (GraphPad, San Diego, CA). All data are expressed as the mean ± standard error mean (SEM) or 95% confidence interval (CI). Statistical comparisons between the groups were performed using one-way repeated measures ANOVA with Tukey's* post hoc* test. Values of *P* < 0.05, 0.01, and 0.001 were considered statistically significant.

## 3. Result

### 3.1. Body Weight and Blood Glucose Level in Normal, DM, and DM-DA Groups

We measured body weights and blood glucose levels in normal, DM, and DM-DA groups. Mean body weight (BW) of normal mice was 30.75 g (95% CI, 29.91–31.59) and blood glucose level (BGL) was 133.83 mg/dL (95% CI, 129.98–137.68). However, BW of DM mice decreased to 26.71 g (95% CI, 25.95–27.47) and BGL increased to more than 600 mg/dL. Also, BW of the groups treated with DA9801 (DM-DA) showed decreased values compared to the normal group, ranging to 28.87 g (95% CI, 26.58–31.16) with unchanged BGL (Table 2). Slightly increased values were shown compared to the DM group. Therefore, these results suggest that DA9801 has no effect on body weights and blood glucose levels.

### 3.2. Effect of DA9801 on Auditory Function

The hearing thresholds in the DM group of the animals assigned to the evaluation of the auditory function show increased values after 8 weeks of treatment compared to normal group, from 12.5 dB (95% CI, 7.85–17.15) to 68.33 dB (95% CI, 64.2–72.46) (Figure 1(a)). However, hearing thresholds in the DM-DA group showed decreased values, 47.5 dB (95% CI, 45.95–49.05), compared to the DM group (Figure 1(a)). DM mice presented delayed wave I–IV latencies compared to the normal group, from 2.79 ms (95% CI, 2.77–2.81) to 3.31 ms (95% CI, 3.05–3.57). On the other hand, wave I–IV latencies of DM-DA group were similar to the normal group by 2.69 ms (95% CI, 2.6–2.78) (Figure 1(b)).

AMLR Pa latencies in DM mice show slower values compared to the normal mice, 23.25 ms (95% CI, 22.3–24.2) to 30.48 ms (95% CI, 29.86–31.1). However, in DA9801 treated group (DM-DA), Pa latencies, 23.58 ms (95% CI, 23.29–23.87), show faster values compared to the DM group (Figure 1(c)). After baseline comparison of ABR and AMLR within groups, no significant differences were found with the animal groups at the beginning of the study (data not shown). These data indicate that DA9801 suppresses the hearing threshold shifts and auditory pathway conduction delay in the diabetic mouse.

### 3.3. Nerve Growth Factor (NGF) Levels in Serum and Sciatic Nerves

In serum and sciatic nerves, NGF expressions of DM groups significantly reduced compared to the normal group. However, NGF ratios of DM-DA groups significantly increased (Figures 2(a) and 2(b)). These data show that DA-9801 endogenously increased NGF level in serum and sciatic nerve.

### 3.4. Nr3c1 Expression in Liver by DA9801

Nr3c1 mRNA expression in the liver showed no change in normal, DA100, and DA300 groups (Figure 3(a)). Unlike mRNA, protein expression of Nr3c1 significantly increased in DA100 and DA300 group in a dose dependent manner (Figure 3(b)). Consequently, DA9801 elevates the systemic Nr3c1 expression.

### 3.5. Tyrosine Kinase A (TrkA) mRNA Expression by DA9801

In DA100 and particularly DA300 group, TrkA levels showed increased expression in a dose dependent manner (Figure 4). These data indicate that DA9801 elevates the systemic TrkA expression.

### 3.6. DA9801 Aggrandize Cell Survival Signal

DA9801 increased p-Akt protein level and significantly changed in DA100 and DA300 groups (Figure 5). As a result, cell survival rate was increased by DA9801 through increased NGF level.

## 4. Discussion

DM may induce hearing impairment through loss of OHCs, spiral ganglion neuron atrophy [2–7], and decreased NGF levels [38, 39]. Previous studies have used neurotrophin, such as a NGF injection method, for overcoming diabetic neuropathy [36, 37]. A different approach based on endogenous NGF has been proposed by DA9801 extract and its mechanism needs to be addressed to understand its applications [41–44].

In this study, we investigated the effect of DA9801 on diabetic hearing impairment and mechanisms of induction of NGF through Nr3c1. This comprehensive study shows that increased ABR thresholds in response to clicks, having delayed ABR waves I–IV latencies and Pa latencies in AMLR, in the presence of auditory function being deteriorated by DM, could be a result of DA9801 treatment. Previous reports have shown that diabetic auditory dysfunction involves alterations in the auditory nerve and central auditory pathway, making electrophysiological tests, such as ABR and AMLR, useful tools for the evaluation of auditory impairments by measurement of hearing thresholds, latencies of waves I–IV, and Pa latency in STZ-induced diabetic animal models and human patients with diabetic neuropathy [8–10].

The ameliorative effects on auditory function shown by DA9801 were accompanied by the NGF release in serum and sciatic nerve. In previous studies, NGF levels have also shown increased value after DA9801 treatment [42], suggesting that this extract induces NGF release in nerves resulting in a physiological recovery and protection of the nerve. However, other mechanisms of DA9801 might be involved in the effects elicited by NGF. Many reports have shown signals related to NGF when it binds with the TrkA receptor such as phosphorylation that sends a signal downstream, and thus Akt transforms to phospho-Akt, resulting in increased cell survival [16–27]. Our results show that mRNA relative levels of TrkA were not changed among the 3 groups, and hence DA9801 has no effect on the transcript of TrkA receptor. However, DA9801 significantly increased phospho-Akt level. This partial relationship with NGF was confirmed with significantly increased Nr3c1 values in the liver after DA9801 treatment. These results suggest that the ameliorative effects of DA9801 showed in the auditory pathways might not involve TrkA receptor. Instead the mechanism of action might be related to elevated neuronal cell survival through elevating Nr3c1, Phospho-Akt, and NGF. In this regard, glucocorticoids have been widely used in the therapy of inner ear disease and acute noise-induced hearing loss [45] and since Nr3c1 is a glucocorticoid receptor found in rat, mouse, and human, even during development stage in mouse ears [46–49], DA9801 might involve this valuable endogenous target. In addition, based on the chemical constituents of the extract, Nr3c1 was found as a biomarker candidate for correlation with NGF and DA9801 using an* in silico* method (data not shown). Therefore, we suggest that DA9801 ameliorates the auditory dysfunction produced by DM through Nr3c1 expression, and thus it induces NGF expression. However, since this study proved the systemic effect of DA9801 in part of the mechanism, further work is needed to investigate the effect on the auditory system and to explore the causal relationships between these biological markers.

## 5. Conclusion

The findings of this study show that recovery effect of DA9801 in the hearing impairment produced by DM model could be elicited by inducing NGF expression through Nr3c1 protein expression via Akt transformation.

## Figures and Tables

**Figure 1:** Hearing thresholds and wave latencies measured by auditory brainstem response (ABR) test, and Pa latencies measured by auditory middle-latency response (AMLR) in normal, DM, and DM-DA groups. (a) Hearing thresholds and (b) wave I–IV latencies by the click stimulus in ABR test of 3 groups. (c) Pa latencies by the click stimulus in AMLR test. ^*^ *P* < 0.05 and ^**^ *P* < 0.01 indicate significant differences from DM group using one-way ANOVA.

**Figure 2:** Nerve growth factor concentrations in serum and sciatic nerves. (a) Nerve growth factor relative ratio in serum and (b) sciatic nerves in normal, DM, and DM-DA groups. ^*^ *P* < 0.05 and ^***^ *P* < 0.001 indicate significant differences from DM group using one-way ANOVA.

**Figure 3:** Nr3c1 mRNA and protein expressions in liver. (a) Immunoblotting was performed on liver protein extracts using antibody of Nr3c1 and *β*-actin which was used as constitutive control for normalization. (b) mRNA levels of Nr3c1 in liver. (c) Relative protein expression levels of Nr3c1. Normal: nondiabetic mice model, DA100: nondiabetic mice model treated with DA9801 100 mg/kg, and DA300: nondiabetic mice model treated with DA9801 300 mg/kg. ^**^ *P* < 0.01 indicates significant differences from normal group using one-way ANOVA.

**Figure 4:** TrkA receptor expressions in liver. There is qPCR analysis of TrkA mRNA expressions in liver. ^**^ *P* < 0.01 indicates significant differences from normal group using one-way ANOVA.

**Figure 5:** p-Akt level in liver. Immunoblotting proves p-Akt level in liver. *β*-actin is reference protein for normalization. Bar graph display normalization of immunoblotting. ^*^ *P* < 0.05 and ^**^ *P* < 0.01 indicate significant differences from normal group using one-way ANOVA.

**Table 1:** Real-time PCR primer sequence.

Gene	Stand	Sequence (5′-3′)	Gene bank accession number
Nr3c1 (glucocorticoid receptor)	Forward	GTG TGA GTC CTT AGT GAC GAG	NM_008173.3
	Reverse	AAG AAG GAG CAA AAT ACT GGG	

TrkA (tyrosine kinase receptor)	Forward	ACC CTT TTG AGT TCA ACC CTG	NM_001033124.1
	Reverse	TCT CTT GAT GTG CTG TTA CCG	

*β*-actin	Forward	TGT ATG AAG GCT TTG GTC TCC	NM_007393.3
	Reverse	GTC TCA AGT CAG TGT ACA GGC	

**Table 2:** Body weights and blood glucose levels of normal, DM, and DM-DA groups.

Groups	Body weight (g)	Glucose levels (mg/dL)
Normal	30.75 ± 1.35	133.83 ± 6.21
DM	26.71 ± 1.22	≥600.00
DM-DA	28.87 ± 3.69	≥600.00

Body weights and blood glucose levels at 8 weeks after DA9801 treatments in normal, DM, and DM-DA groups (normal: nondiabetic mice, DM: STZ-induced diabetic mice model, and DM-DA: STZ-induced diabetic mice were treated with DA9801). The data shown indicate the means ± SEM.
